# Silencing of hsa_circ_0004771 inhibits proliferation and induces apoptosis in breast cancer through activation of miR-653 by targeting ZEB2 signaling pathway

**DOI:** 10.1042/BSR20181919

**Published:** 2019-05-17

**Authors:** Rong Xie, Jing Tang, Xianmin Zhu, Hui Jiang

**Affiliations:** Department of Oncology, Hubei Cancer Hospital, Wuhan 430079, China

**Keywords:** apoptosis, breast cancer, circRNA, miR-653, ZEB2

## Abstract

**Background:** Circular RNAs (circRNAs) have been reported as the competing endogenous RNAs (ceRNAs) to sponge microRNAs (miRNAs) implicating in the initiation and progression of breast cancer. However, the functions of circRNAs in breast cancer have not been completely clarified. In the present study, we aimed to identify differentially expressed circRNAs in breast cancer tumor tissues, and their roles and downstream targets were investigated in the progression of breast cancer. **Methods:** High-throughput circRNA sequencing was performed to detect the differentially expressed circRNAs. The CCK-8 and flow cytometry were performed to measure the cell viability and apoptosis in breast cancer cells. Gene and protein expression were assayed by reverse transcription-quantitative polymerase chain reaction (RT-qPCR) and Western blotting, respectively. **Results:** hsa_circ_0004771 and Zinc finger E-box binding homeobox 2 (ZEB2) expression levels were up-regulated and positively correlated in breast cancer tumor tissues. In addition, the expression levels of miR-653 were reduced in breast cancer tumor tissues. We also found that hsa_circ_0004771 functioned as a sponge of miR-653 to inhibit its expression. miR-653 as a post-transcriptional regulator down-regulated the expression of ZEB2 by binding to its 3′-UTR. Interestingly, a significant inverse correlation was observed between miR-653 and hsa_circ_0004771 or ZEB2 expression in breast cancer tumor tissues. Knockdown of hsa_circ_0004771 and ZEB2 served as equally authentic of miR-653 mimics to induce growth inhibition and apoptosis in breast cancer cells. **Conclusion:** Hsa_circ_0004771/miR-653/ZEB2 regulatory feedback revealed a new molecular mechanism in the pathogenesis of breast cancer, which might provide novel therapeutic targets for the treatment of breast cancer.

## Introduction

Circular RNAs (circRNAs) as a class of endogenous noncoding RNA are predominantly generated in eukaryotes from four cyclized models, including back-spliced exons, circular intronic RNAs, exon–intron circRNAs and intergenic circRNAs and characterized by single-stranded, covalently closed circular molecules without 5′–3′ polarity and polyadenylated tail, reflecting that circRNAs can tolerate the digestion of exonucleases [1,2]. More recently, there have been a growing number of publications focusing on the roles of circRNAs in the pathogenesis of malignancies, such as hepatocellular carcinoma (HCC) [3], gastric cancer [4], non-small-cell lung cancer (NSCLC) [5] and breast cancer [6]. Particularly, with the development of high-throughput sequencing technology and microarray assay, numerous differentially expressed circRNAs are identified in tumor tissues [7,8], while the underlying molecular mechanisms of circRNAs in the carcinogenesis of malignant tumor need yet to be uncovered.

Functional studies have been validated that circRNAs perform multiple functions, including the competing endogenous RNAs (ceRNAs) to sponge microRNAs (miRNAs), interaction with RNA-binding proteins to regulate cell cycle and proliferation and the management of gene transcription and protein translation [9–13]. The canonical function of circRNAs is the miRNAs sponge to recruitment and inactivation of miRNAs, resulting in increased levels of miRNAs targets [9]. For example, circRNA ciRS-7 harbors more than 70 selectively conserved miRNA target sites of miR-7 [9]. In addition, circRNA-SRY contains 16 conserved binding sites of miR-138 and can suppress miR-138 expression and regulate its downstream targets [14]. Notably, some circRNAs, such as circEPSTI1, circIRAK3 and circGFRA1, act as ceRNAs participating in the development and progression of breast cancer by sponging miR-4753 and miR-6809, miR-3607 and miR-34a [6,15,16]. A comprehensive study based on circRNA microarray analysis reveals that more than 1000 circRNAs are deregulated in breast cancer tumor tissues [17]. However, the functions of circRNAs have not been completely clarified in the carcinogenesis of breast cancer.

Zinc finger E-box binding homeobox 2 (ZEB2) is a member of the ZEB family and is constituted by two zinc finger clusters and a central repression region [18]. ZEB2 is originally defined as a transcription factor and executes epithelial-to-mesenchymal transition (EMT) procedures in embryonic development and cancer [19,20]. ZEB2 exhibits a considerable level in various human tumor tissues, including NSCLC [19], HCC [21] and gastric cancer [22]. ZEB2-induced the up-regulation of mesenchymal tissue markers and down-regulation of epithelial cell markers trigger morphological and phenotypic alterations in normal or cancerous cells, leading to the weakness of cellular adhesion and polarity, which are considered as the early and essential step for invasion and metastasis of cancer cells [23]. Numerous studies also reveal that ZEB2 contributes to breast cancer progression by coordinating EMT [24,25]. Post-transcriptional regulatory mechanism has been shown that miR-30a, miR-155 and miR-200 family members inhibit human breast cancer cells invasion by down-regulating ZEB2 [26,27]. However, the association between circRNA and ZEB2 in the pathogenesis of breast cancer is still unclear.

In the present study, the expression profile of circRNAs in breast cancer tumor tissues and corresponding nontumorous tissues was examined by high-throughput sequencing, and the results demonstrated that up-regulation of hsa_circ_0004771 was observed in breast cancer tumor tissues and cell lines. Knockdown of hsa_circ_0004771 inhibited cell proliferation and induced apoptosis in breast cancer cell lines. More importantly, hsa_circ_0004771 could bind to miR-653 as an miRNA sponge to increase ZEB2 expression. *In vitro* experiments uncovered that hsa_circ_0004771/miR-653/ZEB2 axis was involved in breast cancer cells proliferation and apoptosis. In collection, these findings indicated that hsa_circ_0004771/miR-653/ZEB2 signaling pathway provided a new perspective for the treatment of breast cancer.

## Materials and methods

### Patients and specimens

Fifty-one pairs of breast cancer tissues and corresponding nontumourous tissues were obtained from patients who underwent surgical operation in the Hubei Cancer Hospital (Wuhan, China) between January 2009 and January 2014. The normal nontumourous tissues were collected with a distance of more than 3 cm from the edge of cancer tissues. All the specimens for histological and pathological detections were rapidly stored in liquid nitrogen for high-throughput RNA sequencing and reverse transcription-quantitative polymerase chain reaction (RT-qPCR) assay. Written informed consent was obtained from all of the participants prior to samples collection. The study was approved by the Ethics Committee of the Hubei Cancer Hospital (Wuhan, China).

### Cell culture

Normal breast epithelial MCF-10A cell and five breast cancer cell lines (T47D, MCF-7, BT549, Hs-578T and MDA-MB-231) were purchased from the Cell Bank of China Academy of Sciences (Shanghai, China). Cells were cultured in Dulbecco’s modified Eagle’s medium (DMEM; Invitrogen, Carlsbad, CA, U.S.A.) with 10% fetal bovine serum (Thermo Scientific HyClone, Beijing, China), 100 U/ml penicillin and 100 mg/ml streptomycin in a humidified incubator (Thermo Fisher Scientifc, Inc., Waltham, MA, U.S.A.), 5% CO_2_, 95% air atmosphere.

### High-throughput RNA sequencing

RNA extraction from tumor tissues and nontumorous tissues was performed using TRIzol reagent (Invitrogen; Thermo Fisher Scientifc, Inc., Waltham, MA, U.S.A.) and preserved at −80°C until use. RNA concentration was measured using NanoDrop ND-2000 (Thermo Fisher Scientific, Wilmington, DE, U.S.A.). Total RNA (approximately 4 μg) from each sample was subjected to the RiboMinus Eukaryote Kit (Qiagen) to eliminate ribosomal RNA. Purified RNAs were treated with RNase R (Epicenter, 40 U, 37°C, 3 h). Subsequently, using the NEBNext® Ultra™ RNA Library Prep Kit, RNA-seq libraries were prepared and subjected to deep sequencing with an Illumina HiSeq 3000 by RiboBio (RiboBio, Co. Ltd., Guangzhou, China). Differentially expressed circRNAs were selected by *P*-value less than 0.001 and |log_2_fold change| ≥ 1, and the analysis methods were performed as previously described [28,29].

### MiRNAs target prediction

We predicted the miR-653-binding sites of hsa_circ_0004771 and ZEB2 using circinteractome (https://circinteractome.nia.nih.gov/) and TargetScan (http://www.targetscan.org/), respectively. *ZEB2* gene can be transcribed to form multiple transcripts. In the present study, we select one representative transcript (transcript_id: ENST00000558170.2) for molecular mechanism study.

### Cell transfection

MCF-7 and MDA-MB-231 cells were transfected with corresponding plasmids for 48 h at 37°C using Lipofectamine 2000 (Invitrogen, Thermo Fisher Scientifc, Inc., Waltham, MA, U.S.A.) according to the manufacturer’s protocol. The small interfering RNA (siRNA) was synthesized by RiboBio (Guangzhou, China). The targeted sequence of the functional si-0004771 and si-circRNA-NC were 5′-GACAGACGGAAGTGTTTGGAT-3′ and 5′-AAGCCGGAGCTTCGTGGAATC-3′, respectively. The targeted sequence of miR-653 mimics and miR-NC were 5′-UUGAAACAAUCUCUACUGAACC-3′ and 5′-GCCAGCCCUGUAAGUCCCGCAU-3′, respectively. Short hairpin RNA (shRNA) was designed to specifically target ZEB2 using shRNA design tools (http://rnaidesigner.thermofisher.com/rnaiexpress/). Using BLAST (http://blast.ncbi.nlm.nih.gov/Blast.cgi), we have verified that the designed shRNA targeted only the ZEB2. Sh-ZEB2 and shRNA-Con were synthesized by GenePharma (Shanghai, China).

### Cell viability

MCF-7 and MDA-MB-231 cells (1 × 10^4^) were seeded in the 96-well plate for 24, 48 and 72 h transfected with si-0004771 or si-circRNA-NC, miR-653 mimics or miR-NC, and sh-ZEB2 or sh-NC. Cells viability was measured using cell counting kit-8 (CCK-8) Cell Proliferation/Viability Assay Kit (Dojindo Japan). Absorbance was recorded at 450 nm using Elx800 Reader (Bio-Tek Instruments Inc., Winooski, VT, U.S.A.).

### Flow cytometry

MCF-7 and MDA-MB-231 cells (1 × 10^4^) were seeded in the 96-well plate and transfected with si-0004771 or si-circRNA-NC, miR-653 mimics or miR-NC, and sh-ZEB2 or sh-NC for 48 h. Cell apoptosis was monitored using Annexinv-FITC/PI apoptosis detection kit (Carlsbad, California, U.S.A.) according to the manufacturer’s protocol. Apoptotic cell proportion was analyzed by flow cytometry (FACScan, BD Biosciences, San Jose, CA, U.S.A.) and calculated by CELL Quest 3.0 software (BD Biosciences).

### Establishment of tumor xenografts in mice

MCF-7 and MDA-MB-231 cells (1 × 10^7^ cells per 0.1 ml) were transfected with si-0004771 or si-circRNA-NC and were then implanted subcutaneously into 4-week-old female nude mice (*n*=6 in each group, Beijing HFK Bio-Technology. Co., Ltd., China). Tumor weight was measured when mice were killed on day 35 after cell implantation. All the experimental protocols were approved by the Animal Care and Use Committee at Hubei Cancer Hospital (Wuhan, China).

### Luciferase reporter assay

The wild-type (WT) and mutant-type (MUT) 3′-UTR of hsa_circ_0004771 and ZEB2 were inserted into the multiple cloning sites of the luciferase expressing pMIR-REPORT vector (Ambion; Thermo Fisher Scientific, Inc.). For the luciferase assay, MCF-7 and MDA-MB-231 cells (1 × 10^5^) were seeded into 24-wells and co-transfected with luciferase reporter vectors containing the WT or MUT 3′-UTR of hsa_circ_0004771 or ZEB2 (0.5 μg) and miR-653 mimics or miR-NC (100 nM) using Lipofectamine 2000 (Invitrogen; Thermo Fisher Scientific, Inc.), according to the manufacturer’s protocol. The luciferase activity was measured using a luciferase reporter assay kit (Promega, Madison, WI, U.S.A.) according to the manufacturer’s protocol.

### RT-qPCR

#### miRNA RT-qPCR

The total RNA was isolated using TRIzol reagent (Invitrogen; Thermo Fisher Scientifc, Inc., Waltham, MA, U.S.A.). miRNA was subsequently reverse-transcribed to cDNA using the miRNA-specific stem-loop reverse-transcription primer (Ribobio, Guangzhou, China). The relative expression levels of miRNA were calculated using the 2^−ΔΔ*C*^_t_ method [30] and normalized to the internal control U6 using miRNA-specific primers (RiboBio, Guangzhou, China). The reaction conditions were performed according to the instructions from Ribobio Co., Ltd with SYBR Green qPCR Mix (Bio-Rad, Hercules, CA).

#### mRNA RT-qPCR

The cDNA was synthesized by reverse transcription reactions with 2 μg of total RNA using Moloney murine leukemia virus reverse transcriptase (Invitrogen; Thermo Fisher Scientific, Inc.) according to the manufacturer’s protocol. RT-qPCR was performed by Applied Biosystems 7300 Real-Time PCR System (Thermo Fisher Scientific, Inc.) with the TaqMan Universal PCR Master Mix (Thermo Fisher Scientific, Inc.). The relative expression levels of mRNA were calculated using the 2^−ΔΔ*C*^_t_ method [30] and normalized to glyceraldehyde 3-phosphate dehydrogenase (GAPDH). The primers were synthesized by Sangon Biotech (Shanghai, China) as follows: ZEB2: forward primer 5′-CAAGAGGCGCAAACAAGC-3′ and reverse primer 5′-GGTTGGCAATACCGTCATCC-3′; GAPDH: forward primer 5′-GCACCGTCAAGCTGAGAAC-3′ and reverse primer 5′-TGGTGAAGACGCCAGTGGA-3′.

#### CircRNA RT-qPCR

Divergent primers were designed to amplify the head-to-tail splicing of circRNA using RT-qPCR and was performed by Applied Biosystems 7300 Real-Time PCR System (Thermo Fisher Scientific, Inc.) with the TaqMan Universal PCR Master Mix (Thermo Fisher Scientific, Inc.). The PCR primers were as follows: hsa_circ_0102273: forward primer 5′-AAACGTGAAGAAGAGAGTCGTCA-3′ and reverse primer 5′-TCTTTGGTTCAACTTTTCTCCTTGG-3′; hsa_circ_0004771: forward primer 5′-TCCGGATGACATCAGAGCTAC-3′ and reverse primer 5′-TCAAGTGTGCATCTTCTGGCT-3′; hsa_circ_0102272: forward primer 5′-TAGCAATGGGGAAGCTCAGG-3′ and reverse primer 5′-CTGTACCACGTCATCTTGGCT-3′; hsa_circ_0103021: forward primer 5′-GTCAAGAGGACATCCTCACCTC-3′ and reverse primer 5′-GGGGCTGCTAAGCTGATAGG-3′; hsa_circ_0100213: forward primer 5′-GTTTGCCAGTGATTGGACCAG-3′ and reverse primer 5′-GCTTTGTACCTGCAGATGTTGG -3′. GAPDH was used as the reference gene.

### Western blotting

Proteins were extracted with radioimmunoprecipitation assay (RIPA) buffer (Cat. No: P0013B; Beyotime Institute of Biotechnology, Haimen, China). The concentrations were determined using the Bicinchoninic Acid Kit for Protein Determination (Cat. No: BCA1-1KT; Sigma–Aldrich; Merck KGaA). A total of 50 μg of protein for each sample was separated on a 10% SDS/PAGE gel and transferred to nitrocellulose membranes (Bio-Rad Laboratories, Inc., Hercules, CA, U.S.A.). After blocking with 5% nonfat dry milk at room temperature for 2 h, the membranes were incubated with the primary antibody of ZEB2 (Cat. No: sc-271984; dilution: 1:500; Santa Cruz Biotechnology, Inc., Dallas, TX, U.S.A.) at room temperature for 2 h. β-actin (Cat. No: sc-130065; dilution: 1:2000; Santa Cruz Biotechnology) signals were used to correct for unequal loading. Following three washes with TBST, the membranes were incubated with the appropriate horseradish peroxidase–conjugated secondary antibody (Cat. No: sc-516102; dilution: 1:10000; Santa Cruz Biotechnology) at room temperature for 2 h and visualized by chemiluminescence (Thermo Fisher Scientific, Inc.). Signals were analyzed with Quantity One® software version 4.5 (Bio-Rad Laboratories, Inc., Hercules, CA, U.S.A.).

### Statistical analysis

Data were presented as mean ± standard deviation. Statistical analysis was performed using GraphPad Prism Version 7.0 (GraphPad Software, Inc., La Jolla, CA, U.S.A.). Student’s *t* test was used to analyze two-group differences. Inter-group differences were analyzed by one-way analysis of variance, followed by Tukey’s post hoc analysis. Survival analysis was performed using the Kaplan–Meier method with the log-rank test applied for comparison. Spearman’s rank analysis was used to identify the correlation between hsa_circ_0004771 and miR-653, or hsa_circ_0004771 and ZEB2 or miR-653 and ZEB2. *P*<0.05 was considered to indicate a statistically significant difference.

## Results

### CircRNAs expression profile in breast cancer tumor tissues and corresponding nontumorous tissues

We first performed high-throughput sequencing to detect circRNAs expression profile in five pairs of breast cancer tumor tissues and corresponding nontumorous tissues. We identified that 49 circRNAs were significantly and differentially expressed between the two groups by screening for the log_2_ fold change more than 1 and *P*-value less than 0.001 (Figure 1A). Among these circRNAs, 30 circRNAs were significantly up-regulated and 19 circRNAs were significantly down-regulated in tumor tissues from breast cancer patients (Figure 1A). To validate the results of high-throughput sequencing, we selected top five circRNAs (hsa_circ_0102273, hsa_circ_0004771, hsa_circ_0102272, hsa_circ_0103021 and hsa_circ_0100213) for further assessment using RT-qPCR, and the findings demonstrated that RT-qPCR results were consistent with sequencing data that top five circRNAs were markedly increased in breast cancer tumor tissues compared with corresponding nontumorous tissues (Figure 1B–F). We summarized the genetic information of top five circRNAs as shown in Figure 1G. We also found that the expression of hsa_circ_0004771 was higher than others four circRNAs (Figure 1G). Therefore, we focused on hsa_circ_0004771 in our further study.

**Figure 1:** CircRNAs expression profile in breast cancer tumor tissues and corresponding nontumorous tissues The cluster heatmap represents significant differentially expressed circRNAs more than two-fold change among five pairs of breast cancer tissues and corresponding nontumourous tissues. Red color indicates high expression level, and green color indicates low expression level (**A**). The expression levels of top five up-regulated circRNAs, including hsa_circ_0102273 (**B**), hsa_circ_0004771 (**C**), hsa_circ_0102272 (**D**), hsa_circ_0103021 (**E**) and hsa_circ_0100213 (**F**), were measured by RT-qPCR assay in 51 pairs of breast cancer tumor tissues and corresponding nontumorous tissues. Furthermore, the biological characteristics of top five up-regulated circRNAs were summarized (**G**). *P<0.05 compared with corresponding nontumorous tissues. Abbreviations: N, nontumorous tissue; T, tumor tissue.

RT-qPCR analysis of hsa_circ_0004771 levels in 51 pairs of breast cancer tumor tissues and corresponding nontumorous tissues indicated that 43 of these cases exhibited the up-regulation of hsa_circ_0004771 in breast cancer tumor tissues (Figure 2A). An analysis of hsa_circ_0004771 expression was carried out among normal breast epithelial MCF-10A cell and five breast cancer cell lines (T47D, MCF-7, BT549, Hs-578T and MDA-MB-231). Surprisingly, up-regulation of hsa_circ_0004771 was observed in five breast cancer cell lines as compared with MCF-10A cell, especially in MCF-7 and MDA-MB-231 cell lines (Figure 2B). Furthermore, Kaplan–Meier analysis was used to investigate the correlation between hsa_circ_0004771 level and overall survival prognosis in breast cancer patients. High and low expression groups were segregated according to Log_2_ fold change ≥ 1. We found that breast cancer patients with high hsa_circ_0004771 levels had a significantly poorer survival prognosis than that in low expression group (Figure 2C).

**Figure 2:** High hsa_circ_0004771 level was associated with poor survival prognosis in breast cancer patients The Log_2_ fold change of hsa_circ_0004771 expression in 51 pairs of breast cancer tumor tissues and corresponding nontumorous tissues was calculated, and the results showed that hsa_circ_0004771 was up-regulated in 43 of 51 breast cancer patients (**A**). An analysis of hsa_circ_0004771 expression was carried out among normal breast epithelial MCF-10A cell and five breast cancer cell lines (T47D, MCF-7, BT549, Hs-578T and MDA-MB-231) (**B**). Kaplan–Meier survival curve was used to evaluate whether hsa_circ_0004771 expression level was associated with overall survival prognosis in breast cancer patients (**C**). *P<0.05; **P<0.01; ***P<0.001 compared with normal control group.

### Knockdown of hsa_circ_0004771 inhibits cell proliferation and induces apoptosis in breast cancer cells

To determine the role of hsa_circ_0004771 on cell proliferation and apoptosis in breast cancer cells, we knocked down hsa_circ_0004771 in MCF-7 and MDA-MB-231 cells, reflecting that the expression of hsa_circ_0004771 was significantly inhibited after transfection with si-0004771 compared with that in si-NC group (Figure 3A). CCK-8 assays showed that hsa_circ_0004771 knockdown led to the inhibition of cell proliferation in MCF-7 and MDA-MB-231 cells (Figure 3B). AnnexinV-FITC apoptosis analysis revealed that hsa_circ_0004771 depletion resulted in the increase in apoptosis rate in MCF-7 and MDA-MB-231 cells (Figure 3C). We next evaluated the effects of hsa_circ_0004771 on MCF-7 and MDA-MB-231 xenografts in mice. After knockdown of hsa_circ_0004771 in MCF-7 and MDA-MB-231 cells, cells were implanted subcutaneously into immune-deficient mice, and tumor growth was monitored for 5 weeks after cell implantation. The results showed that hsa_circ_0004771 silence significantly reduced tumor volume (Figure 3D) and weight (Figure 3E) *in vivo*.

**Figure 3:** Knockdown of hsa_circ_0004771 inhibited cell proliferation and induced apoptosis in breast cancer cells After transfection with si-hsa_circ_0004771 (si-0004771) into MCF-7 and MDA-MB-231 cells, the expression levels of hsa_circ_0004771 were evaluated by RT-qPCR assay (**A**); cell viability was assessed by CCK-8 assay (**B**); cell apoptosis was measured using Annexin V-FITC/PI staining and flow cytometry analysis (**C**). MCF-7 and MDA-MB-231 cells (1 × 10^7^ cells per 0.1 ml) transfected with si-0004771, and then cells implanted subcutaneously into 4-week-old female nude mice (*n*=6 in each group), and tumor volume (**D**) and weight (**E**) was calculated at day 35 after cell implantation. *P<0.05; **P<0.01; ***P<0.001 compared with control group.

### Hsa_circ_0004771 directly targets miR-653

To investigate circRNA–miRNA interaction pathways, bioinformatics databases TargetScan (http://www.targetscan.org/) and circinteractome (https://circinteractome.nia.nih.gov/) were used to predict potential binding sites of miRNAs in hsa_circ_0004771. Our results uncovered that 13 miRNAs had binding sites within hsa_circ_0004771, and 8 miRNAs, including miR-1203, miR-149, miR-532-3p, miR-580, miR-589, miR-595, miR-653 and miR-924, were significantly reduced in breast cancer tumor tissues compared with corresponding nontumorous tissues (Figure 4A), especially miR-653 at the minimum level. Therefore, we paid close attention to miR-653 in our further experiments. Next, Spearman’s rank correlation analysis was used to evaluate the association between hsa_circ_0004771 and miR-653 expression in breast cancer tumor tissues, and the results found that a significant negative correlation between hsa_circ_0004771 and miR-653 was observed in 51 breast cancer tumor tissues (r = −0.719, *P*<0.001; Figure 4B). We also found that low miR-653 expression was associated with poor survival prognosis in breast cancer patients (Figure 4C). To verify miR-653 was a direct target of hsa_circ_0004771, we first delineated the conserved binding sites using online prediction softwares as shown in Figure 4D. Subsequently, luciferase report assay showed that overexpressed miR-653 co-transfected with WT hsa_circ_0004771 segment resulted in significant reduction in fluorescence intensity in MCF-7 and MDA-MB-231 cells (Figure 4E). In contrast, the fluorescence intensity had no significant difference between control group and cells co-transfected with miR-653 and MT hsa_circ_0004771 segment (Figure 4F).

**Figure 4:** Hsa_circ_0004771 directly targeted miR-653 Thirteen miRNAs were predicted to bind with hsa_circ_0004771, and the expression levels of 13 miRNAs were measured by RT-qPCR assay in 51 pairs of breast cancer tumor tissues and corresponding nontumorous tissues (**A**). Spearman’s rank correlation analysis was performed to evaluate the association between hsa_circ_0004771 and miR-653 expression in breast cancer tumor tissues (**B**). Kaplan–Meier survival curve analysis showed that miR-653 low expression was a risk factor for poor prognosis in breast cancer patients (**C**). The putative binding sites between hsa_circ_0004771 and miR-653 were predicted by online softwares (**D**) and verified by luciferase activity reporter assays (**E** and **F**). *P<0.05 compared with normal control group.

### Overexpression of miR-653 inhibits cell proliferation and induces apoptosis in breast cancer cells

Intriguingly, we found that up-regulation of miR-653 was accompanied with reduction in tumor volume and weight in hsa_circ_0004771 silent MCF-7 and MDA-MB-231 xenografts mice (Figure 5A). Therefore, we hypothesized that miR-653 might be a regulator involved in breast cancer cell growth inhibition. We performed *in vitro* experiments to determine the effect of miR-653 on MCF-7 and MDA-MB-231 cell proliferation and apoptosis by transfecting with miR-653 mimics. The expression of miR-653 was significantly elevated in MCF-7 and MDA-MB-231 cell after transfected with miR-653 mimics as compared with in the control group (Figure 5B). As expected, miR-653 gain-of-function inhibited MCF-7 and MDA-MB-231 cells proliferation (Figure 5C) and induced apoptosis (Figure 5D) *in vitro*.

**Figure 5:** Overexpression of miR-653 inhibited cell proliferation and induced apoptosis in breast cancer cells After transfection with si-0004771 into MCF-7 and MDA-MB-231 cells, the expression levels of miR-653 were evaluated by RT-qPCR assay (**A**). After transfection with miR-NC or miR-653 mimics into MCF-7 and MDA-MB-231 cells, the expression levels of miR-653 were evaluated by RT-qPCR assay (**B**); cell viability and apoptosis were measured by CCK8 (**C**) and Annexinv-FITC/PI staining (**D**), respectively. *P<0.05; ***P<0.001 compared with control group.

### ZEB2 is a direct target of miR-653

To investigate whether ZEB2 was a direct target of miR-653, TargetScan was used to predict the potential binding sites of miR-653 in the 3′-UTR of ZEB2. As shown in Figure 6A, the 3′-UTR of ZEB2 contained one conserved binding site of miR-653, which was confirmed by luciferase report assay (Figure 6B,C). We also found that overexpression of miR-653 could suppress ZEB2 protein expression in MCF-7 and MDA-MB-231 cells (Figure 6D). The mRNA expression of ZEB2 was increased in breast cancer tumor tissues (Figure 6E), which was inversely correlated with miR-653 expression (Figure 6F).

**Figure 6:** ZEB2 was a direct target of miR-653 The putative binding sites between ZEB2 and miR-653 were predicted by online softwares (**A**) and verified by luciferase activity reporter assays (**B** and **C**). After transfection with miR-NC or miR-653 mimics into MCF-7 and MDA-MB-231 cells, the protein expression levels of ZEB2 were measured by Western blotting (**D**). The mRNA expression levels of ZEB2 were measured by RT-qPCR in 51 pairs of breast cancer tumor tissues and corresponding nontumorous tissues **(E**). Spearman’s rank correlation analysis was performed to evaluate the association between ZEB2 mRNA expression and miR-653 expression in breast cancer tumor tissues (**F**). *P<0.05; ***P<0.001 compared with control group.

### Knockdown of ZEB2 inhibits cell proliferation and induces apoptosis in breast cancer cells

To explore the effect of ZEB2 on MCF-7 and MDA-MB-231 cell proliferation and apoptosis, shRNA was transfected into MCF-7 and MDA-MB-231 cells to inhibit the mRNA expression of ZEB2 (Figure 7A). There was a significant decrease in cell proliferation (Figure 7B) and increase in apoptosis rate (Figure 7C) in MCF-7 and MDA-MB-231 cells transfected with sh-ZEB2. In MCF-7 xenografts mice with hsa_circ_0004771 knockdown, the mRNA and protein expression of ZEB2 were decreased in solid tumor (Figure 7D,E). We also found that the mRNA expression of ZEB2 was positively related with hsa_circ_0004771 expression in breast cancer tumor tissues (Figure 7F). Furthermore, Kaplan–Meier survival curve analysis revealed that high expression of ZEB2 was closely related with poor prognosis in patients with breast cancer (Figure 7G).

**Figure 7:** Knockdown of ZEB2 inhibited cell proliferation and induced apoptosis in breast cancer cells After transfection with sh-NC or sh-ZEB2 into MCF-7 and MDA-MB-231 cells, the mRNA expression levels of ZEB2 were measured by RT-qPCR assay (**A**) cell viability and apoptosis were measured by CCK8 (**B**) and Annexin V-FITC/PI staining (**C**) respectively. After transfection with si-NC or si-0004771 into MCF-7 and MDA-MB-231 cells, the mRNA (**D**) and protein (**E**) expression levels of ZEB2 were measured by RT-qPCR and Western blotting assay, respectively. Spearman’s rank correlation analysis was performed to evaluate the association between ZEB2 mRNA expression and hsa_circ_0004771 expression in breast cancer tumor tissues (**F**). Kaplan–Meier survival curve analysis showed that ZEB2 high expression was a risk factor for poor prognosis in breast cancer patients (**G**). *P<0.05; ***P<0.001 compared with control group.

## Discussion

In our study, hsa_circ_0004771 and ZEB2 expression levels were up-regulated and positively correlated in breast cancer tumor tissues. We also found that hsa_circ_0004771 functioned as a sponge of miR-653 to inhibit its expression. miR-653 as a post-transcriptional regulator down-regulated the expression of ZEB2 by binding to its 3′-UTR. Interestingly, a significant inverse correlation was observed between miR-653 and hsa_circ_0004771 or ZEB2 expression in breast cancer tumor tissues. Knockdown of hsa_circ_0004771 and ZEB2 served as the equally authentic of miR-653 mimics to induce growth inhibition and apoptosis in breast cancer cells. In summary, hsa_circ_0004771/miR-653/ZEB2 regulatory feedback revealed a new molecular mechanism in the pathogenesis of breast cancer, which might provide novel therapeutic targets for the treatment of breast cancer.

Numerous studies have been proven that circRNAs as miRNAs sponge and ceRNA result in reduced miRNAs activity and elevated levels of miRNAs-targeted transcripts [1,9,10]. Some circRNAs, including hsa_circ_0072995, hsa_circ_0052112, circIRAK3 and circGFRA1 promotes breast cancer cell migration and invasion by sponging miR-30c-2-3p, miR-3607 miR-125a-5p and miR-34a expression, respectively [15,16,31,32]. These findings coincide with our conclusion that hsa_circ_0004771 can serve as a ceRNA to inhibit miR-653 expression in breast cancer tumorigenesis. Intriguingly, Lü et al. validates a significant up-regulation of hsa_circ_0004771 expression levels in breast cancer tumor tissues and demonstrates that hsa_circ_0004771 and its target hsa-miR-339-5p may be associated with the carcinogenesis of breast cancer [17].

miR-653-5p and miR-653-3p are the mainly subtypes of miR-653, miR-653-5p targets 615 transcripts with conserved sites, containing a total of 662 conserved sites and 487 poorly conserved sites, and miR-653-3p regulates 4960 transcripts with very poorly conserved sites, containing a total of 6832 sites (TargetScan, www.targetscan.org). miR-653 has been reported to exert regulatory functions in mammalian evolution [33,34]. However, the functions of miR-653 in the regulation of cancer progression have on relevant report. In the present study, miR-653 expression was reduced in breast cancer tissues, and breast cancer patients with miR-653 low expression associated with poor survival prognosis. Moreover, miR-653 was identified as a tumor suppressor due to its suppression of the ZEB2 expression.

Overexpression of ZEB2 is implicated in various malignant carcinomas, reflecting that ZEB2 promotes tumor metastasis, invasiveness and correlates with poor prognosis of human colorectal cancer, glioma, acute myeloid leukemia and small cell lung cancer [19,35–38]. Both up-regulation of ZEB2 and down-regulation of E-cadherin enhance the EMT, which results in increased migration and invasion in MCF-7 and MDA-MB-231 cells [39]. Moreover, ZEB2 plays a synergistic effect with cdc42 GTPase-activating protein, as a novel E-cadherin transcriptional repressor, to facilitate breast cancer tumor growth and metastasis to lung [40]. Previous studies also uncover that ZEB2 can be regulated by miRNAs, including miR-29b, miR-30a, miR-155, miR-204 and miR-205, in the development of breast cancer aggressiveness [26,27,39,41,42]. In the present study, our findings extended the role of ZEB2, as an oncogene promotion of cell proliferation in breast cancer, that was a direct target of miR-653. A significant negative correlation between ZEB2 and miR-653 expression was observed in breast cancer tissues. ZEB2 played a completely opposite role to miR-653 in survival prognosis, cell proliferation and apoptosis. Among these candidate miRNAs, we also found that algorithms predicted ZEB2 was a target of miR-532-3p. Based on the expression of miR-653 was lower that miR-532-3p in the breast cancer tissues, our study mainly focused on the functions of miR-653 in the progression of breast cancer. Although we could not fully expound the roles of miR-532-3p in the present study; we guaranteed that the underlying molecular mechanisms of miR-532-3p will be explored in our future research.

In conclusion, our findings suggested that miR-653 was able to target both hsa_circ_0004771 and ZEB2, reflecting that hsa_circ_0004771 might serve as miR-653 sponge to modulate ZEB2 expression through the ceRNA mechanism. Bioinformatics prediction and luciferase reporter assays verified these conclusions. We also found that hsa_circ_0004771 performed a parallel effect to ZEB2 and an opposite effect to miR-653 in breast cancer cell proliferation and apoptosis. More importantly, hsa_circ_0004771/miR-653/ZEB2 aixs contributed to the development of the new therapeutic targets for the treatment of breast cancer.

## Compliance with ethical standards

The study was approved by the Ethics Committee of the Hubei Cancer Hospital (Wuhan, China). Written informed consent was obtained from all of the participants prior to sample collection.

## Abbreviations

CCK-8: cell counting kit-8
ceRNA: competing endogenous RNA
circRNA: circular RNA
EMT: epithelial-to-mesenchymal transition
GAPDH: glyceraldehyde 3-phosphate dehydrogenase
HCC: hepatocellular carcinoma
miRNA: microRNA
MUT: mutant-type
NSCLC: non-small-cell lung cancer
RT-qPCR: reverse transcription-quantitative polymerase chain reaction
TBST: tris buffered saline tween
WT: wild-type
ZEB2: Zinc finger E-box binding homeobox 2
